# Establishment and Validation of a Machine Learning Prediction Model Based on Big Data for Predicting the Risk of Bone Metastasis in Renal Cell Carcinoma Patients

**DOI:** 10.1155/2022/5676570

**Published:** 2022-10-03

**Authors:** Chan Xu, Wencai Liu, Chengliang Yin, Wanying Li, Jingjing Liu, Wanli Sheng, Haotong Tang, Wenle Li, Qingqing Zhang

**Affiliations:** ^1^Department of Dermatology, Xianyang Central Hospital, Xianyang 712000, China; ^2^Department of Clinical Medical Research Center, Xianyang Central Hospital, Xianyang 712000, China; ^3^Department of Orthopaedic Surgery, The First Affiliated Hospital of Nanchang University, Nanchang 330006, China; ^4^Faculty of Medicine, Macau University of Science and Technology, Macau 999078, China; ^5^Department of Shanghai National Engineering Research Center of Biochip, Shanghai 201203, China; ^6^Hohhot Technical Center of Hohhot Customs District, Hohhot 010020, China; ^7^Molecular Imaging and Translational Medicine Research Center, State Key Laboratory of Molecular Vaccinology and Molecular Diagnostics, Xiamen University, Xiamen 361005, China; ^8^Department of Otolaryngology-Head and Neck Surgery, The Second Affiliated Hospital of Xi'an Jiao Tong University, Xi'an 710004, China

## Abstract

**Purpose:**

Since the prognosis of renal cell carcinoma (RCC) patients with bone metastasis (BM) is poor, this study is aimed at using big data to build a machine learning (ML) model to predict the risk of BM in RCC patients.

**Methods:**

A retrospective study was conducted on 40,355 RCC patients in the SEER database from 2010 to 2017. LASSO regression and multivariate logistic regression analysis was performed to determine independent risk factors of RCC-BM. Six ML algorithm models, including LR, GBM, XGB, RF, DT, and NBC, were used to establish risk models for predicting RCC-BM. The prediction performance of ML models was weighed by 10-fold cross-validation.

**Results:**

The study investigated 40,355 patients diagnosed with RCC in the SEER database, where 1,811 (4.5%) were BM patients. Independent risk factors for BM were tumor grade, T stage, N stage, liver metastasis, lung metastasis, and brain metastasis. Among the RCC-BM risk prediction models established by six ML algorithms, the XGB model showed the best prediction performance (AUC = 0.891). Therefore, a network calculator based on the XGB model was established to individually assess the risk of BM in patients with RCC.

**Conclusion:**

The XGB risk prediction model based on the ML algorithm performed a good prediction effect on BM in RCC patients.

## 1. Introduction

Renal cell carcinoma (RCC), a renal space-occupying lesion originating from renal tubular epithelial cells, accounts for 4% of all malignant tumors [1]. As the most common type of renal cancer, RCC took up 85%-90% of renal malignant tumors in adults [2]. Since the early clinical manifestations of RCC are hidden, 20%-40% of patients will eventually suffer from metastatic RCC (mRCC) [3]. At present, surgical resection is the first-line treatment for RCC. However, in some RCC patients, distant metastasis after radical nephrectomy still reappeared or even occurred [4]. In addition, most RCC will become resistant to chemotherapy and radiotherapy once they develop into relapse or metastasis [5].

Bone metastasis (BM) is one of the most frequent sites of solid malignant tumors, the occurrence of which reveals the poor prognosis of tumor patients. As RCC has obvious osteotaxis in distant metastasis, bone is the second common distant metastasis site of RCC except the lung [6, 7]. Studies have shown that in about 20-35% of patients with RCC disease progression, renal cell carcinoma bone metastasis (RCC-BM) will emerge, such as the pelvis, spine, and ribs [3]. BM of RCC mainly leads to osteolytic destructive changes such as skeletal-related events (SER) [8], including pathological fracture, spinal cord and/or nerve root compression, and bone pain [9]. More than 70% of BM-RCC patients have experienced at least one SER during their survival, which severely reduced their quality of life and survival time [10]. Previous studies indicated that the prognosis of patients with RCC-BM was poor. Their median overall survival time (OST) was only 12-28 months, and the 5-year overall survival rate was only 11%, while the median OST of mRCC patients without BM was prolonged to 31 months and the 5-year overall survival rate increased to 47% [10, 11]. Therefore, bone metastasis is an important cause of death in patients with advanced RCC and it is crucial to predict the risk of RCC-BM.

Several previous studies reported the risk factors and prognostic factors of BM in RCC patients [12–15], and some developed traditional nomograms to predict the risk of RCC-BM [5]. However, there are few studies using machine learning (ML) method to construct the risk prediction model of RCC-BM based on big data. This study is aimed at (1) setting up the RCC-BM risk prediction model through ML and verifying the validity of the model with external data and (2) constructing a network calculator to facilitate clinicians to choose more reasonable diagnosis and treatment for RCC patients.

## 2. Methods

### 2.1. Study Population Selection

The training group data analyzed in this study are from the SEER database (http://seer.cancer.gov/about/), where the analysis of anonymous data is exempt from medical ethics review and does not require informed consent from patients.

### 2.2. Data Collection

All RCC data in the retrospective cohort study from 2010 to 2017 were extracted and subsumed as training group data with SEER∗Stat (version 8.3.6) software. According to the inclusion/exclusion criteria, 40,355 patients were selected into the training group. The inclusion/exclusion criteria were as follows: (1) RCC was the first or primary tumor; (2) patients with RCC diagnosed by pathology (the validation group was diagnosed by at least two pathologists blindly); (3) patients with complete clinicopathological features, demographic data, and follow-up data; and (4) patients with RCC proved by autopsy or death were excluded from this study.

Based on the specific information of RCC patients from the SEER database, 17 variables were selected to determine the independent risk factors of BM in RCC patients, including marital status, age, race, serial number, survival time, survival status, gender, primary location, grade, side, pathological stage, T stage, N stage, tumor size, bone metastasis, brain metastasis, and liver metastasis. The risk prediction models were framed using data of the training group.

### 2.3. Establishment and Verification of Prediction Models

Six ML models, including logistic regression (LR), gradient boosting machine (GBM), extreme gradient boosting (XGB), Random Forest (RF), Decision Tree (DT), and Naive Bayesian model (NBC), were used to build prediction models, the performance of which was compared by 10-fold cross-validation method [16–19]. The model with the greatest AUC value was regarded as the preferred prediction model, whose corresponding network calculator is designed to individually assess the risk of BM in patients with RCC [20–23].

### 2.4. Statistical Analysis

The measurement data is expressed in mean (SD), and the counting data is expressed in frequency (percentage). Independent samples *t*-test, chi-square test, LASSO regression analysis, univariate and multivariate logistic regression analysis, 10-fold cross-validation, and other statistical analysis were performed by SPSS 26.0 (SPSS Inc., Chicago, USA) software. *P* values < 0.05 were considered statistically significant. R software (version 4.0.5, https://www.r-project.org/) was applied for drawing the correlation heat map and ROC curve and developing a predictive model which used the “shiny” package to establish a web calculator.

## 3. Results

### 3.1. Characteristics of the Study Population

A total of 40,355 RCC patients from the SEER database were included in this study to establish the training group. 4.5% (1811 cases) of RCC patients progressed to BM. Then, six risk factors for predicting BM in RCC patients were screened by LASSO regression, including tumor grade, T stage, N stage, liver metastasis, lung metastasis, and brain metastasis (Figure 1), which were viewed as predictors in the correlation heat map (Figure 2).

### 3.2. Independent Risk Factors of BM in RCC Patients

Univariate and multivariate logistic regression analyses were carried out to value the independent risk factors of BM in RCC patients. Univariate logistic regression analysis displayed that brain metastasis, liver metastasis, lung metastasis, tumor grade, T stage, and N stage were importantly associated with BM in patients with RCC (*P* < 0.05). Further multivariate logistic regression analysis indicated that brain metastasis (OR = 2.46, 95%CI = 1.98 − 3.05), liver metastasis (OR = 2.37, 95%CI = 2.01 − 2.8), lung metastasis (OR = 5.2, 95%CI = 4.58 − 5.89), tumor grade (poorly differentiated: OR = 3.08, 95%CI = 1.87 − 5.08; undifferentiated: OR = 4.47, 95%CI = 2.69 − 7.42; undifferentiated: OR = 7.97, 95%CI = 4.9 − 12.97), T stage (T2 stage: OR = 2.13, 95%CI = 1.81 − 2.5; T3 stage: OR = 1.84, 95%CI = 1.59 − 2.13; T4 stage: OR = 2.08, 95%CI = 1.68 − 2.59; and TX stage: OR = 3.11, 95%CI = 2.51 − 3.86), and N stage (N1 stage: OR = 2.18, 95%CI = 1.9 − 2.51; NX stage: OR = 1.64, 95%CI = 1.34 − 2.01) were independent risk factors for BM in RCC patients (*P* < 0.001, Table 1).

### 3.3. Selection and Verification of the Prediction Models

The prediction performance of six ML algorithm models (LR, NBC, DT, RF, GBM, and XGB) was compared by 10-fold cross-validation method, which indicates that the prediction value of all models above was great (AUC > 0.850). In descending order, the predictive ability of models is XGB, RF, GBM, NBC, LR, and DT, of which XGB is the best in predicting RCC-BM (average AUC = 0.891, Figure 3). Therefore, the XGB model is selected as the optimal prediction model finally.

The importance of each risk factor is not identical in different ML prediction models. Among them, lung metastasis is the most important clinical feature in the six models, while brain metastasis is of the least significance feature in RF, GBM, and XGB models, familiar as tumor grade in NBC and DT models and N stage in the LR model. In the XGB model, the independent risk factors are arranged according to their importance, which are lung metastasis, T stage, liver metastasis, tumor grade, N stage, and brain metastasis. The value of risk factors in other models is shown in Figure 4.

### 3.4. Construction of the Web Calculator

Based on the GBM model possessing the best performance, a risk web calculator was designed in this study (https://share.streamlit.io/liuwencai5/renal_bone/main/renal_bone.py). By inputting the relevant clinicopathological variables of RCC patients, clinicians could predict the risk of BM in patients with RCC (Figure 5).

## 4. Discussion

As an important marker of poor prognosis in patients with RCC, early detection and intervention for BM are urgently needed. Guo et al. [14] analyzed the data of 45,824 RCC patients recorded in the SEER database from 2010 to 2014 and found that 3.29% patients were diagnosed with BM at the initial diagnosis. In our study, 4.5% RCC patients in the training group developed into BM, while Zekri et al. [24] reported that 30-40% of advanced RCC patients turned into BM. Therefore, the incidence rate of BM may be underestimated since the patients showed no symptoms when the initial diagnosis was made or BM appeared at the advanced stage of RCC disease which was not recorded in the SEER database. At present, the guidelines only recommend bone imaging for patients with uncomfortable symptoms or abnormal alkaline phosphatase level [25]. Thus, consequently, patients with asymptomatic BM could not be treated timely and effectively. At present, bone metastasis has been recognized as one of the adverse prognostic factors of RCC patients [8]. In addition, the resection of whole spinal BM can prolong the survival time potentially for the patients with isolated spinal BM and no visceral metastasis [26], but the prognosis of BM in RCC patients is still poor compared with that of other tumors such as lung cancer. With the improved bone-targeted therapy of BM patients, the average OST of BM patients is 12.0-31.8 months [27–29]. The lack of effective chemotherapeutic drugs may be the main reason for the poor outcome of RCC patients with BM [11]. Due to the occult onset and poor prognosis of BM, it is necessary to study the risk factors of BM in patients with RCC. Additionally, early identification and evaluation of BM are of great significance to improve the precision of the diagnosis, determine the treatment plans, and prevent RCC complications such as SER in patients with symptomless BM.

In this study, multivariate logistic regression analysis revealed that brain metastasis, liver metastasis, lung metastasis, poor tumor differentiation, high T stage, and N stage were independent risk factors for BM in RCC patients. Similarly, Guo et al. [14] found that male gender; higher T stage; lymph node involvement; poor tumor differentiation; presence of lung, liver, and brain metastasis; and the collecting duct type of RCC were positively associated with BM occurrence. Furthermore, Fan et al. [30], using nomogram to quantify the risk of RCC-BM patients, found that the independent factors of RCC complicated with BM include grade, histological type, N stage, operation, brain metastasis, and lung metastasis, which was basically consistent with our research results. Additionally, through a retrospective analysis of 372 RCC patients, Chen et al. [31] discovered that the concentrations of ALP, calcium, and Hb were potential risk factors for bone metastasis in patients with RCC. ALP > 105.5 U/L,calcium > 2.615 mmol/L, andHb < 111.5 g/L in newly diagnosed RCC patients suggest that BM is more likely to occur in these patients; hence, close monitoring and active bone scanning should be carried out to determine whether bone metastasis has happened. With the in-depth study of RCC-BM, more and more prognostic factors of bone metastasis also have been discovered. Yoshiyama et al. [32] considered that patients' age, ECOG performance, histology, MSKCC prognosis score, concomitant metastasis, and the time from nephrectomy to bone metastasis were important factors related to the prognosis of RCC-BM. Subsequently, Ruatta et al. [15] tracked 1750 RCC patients and found that MSKCC score, BMs number, and radical resection were essential prognostic factors for RCC patients with BMs.

With the development of TNM staging system and pathological classification criteria of renal cell carcinoma, a variety of RCC prognosis analysis systems have appeared. But they have several limitations. TNM staging system depends on three pathological indexes while it ignores other risk factors, which reduces the accuracy of prognosis prediction of RCC patients. MSKCC model (Memorial Sloan Kettering Cancer Center-based poor-risk groups) and IMDC model (International Metastatic Renal Cell Carcinoma Database Consortium-based poor-risk groups) [27] lack the function of comprehensive analysis for patients. GRCC model (Gustave Roussy Cancer Campus) [33] is more accurate and convenient than the MSKCC and IMDC prognostic analysis model, but it is not designed for RCC-BM patients specifically. The B-FOM scoring system (Fujimoto–Owari–Miyake bone score) is characterized by bone metastasis specificity, yet poor tissue source specificity is its short board [34]. The traditional Cox regression or logistic regression analysis is visualized in this article; thus, clinicians can easily calculate the probability of BM in RCC patients without understanding the complex underlying mathematical formula. Distinguished from prediction analysis system or model mentioned above, this study creatively developed and verified six machine learning algorithms models, which were specially performed to estimate the risk of BM in RCC patients. The XGB model with the best prediction performance was selected through 10-fold verification methods, and an online calculator was established to evaluate the individual probability of RCC-BM. The ML-based model can be used to guide clinical treatment decisions, help clinicians better predict the BM risk, and take necessary interventions to improve the survival time and life quality of RCC patients.

The limitations of our study could not be ignored though. Firstly, as a retrospective cohort study, the inevitable selection bias may affect the results considerably. Since the SEER database only collects the initial diagnosis results, BM arising in the advanced stage of RCC may be omitted. Secondly, the deficiency of external validation using the data from the local validation group patients could not assess the accuracy of the selected XGB models in diagnosing BM in RCC patients and therefore establish the other clinical utility analysis such as probability density functions (PDF) and clinical utility curves (CUC). Additionally, we were unable to obtain some effective indicators for predicting RCC-BM from SEER, such as transforming growth factor-*β* (TGF-*β*) [35], fibroblast growth factor (FGF) [1], insulin-like growth factor [36], bone morphogenetic protein [37], AFP [38], CA-199 [31], and Fuhrman nuclear grade [39]. Future studies are needed to incorporate tumor characteristics, laboratory results, and treatment regimens to establish a higher dimensional predictive model.

## 5. Conclusion

This study retrospectively analyzed the independent risk factors of BM in renal cell carcinoma based on the SEER database, including tumor grade, T stage, N stage, liver metastasis, lung metastasis, and brain metastasis. On the foundation of the SEER dataset, we constructed and validated six machine learning models including LR, GBM, XGB, RF, DT, and NBC and subsequently selected XGB as the optimal prediction model. The network calculator designed on the basis of XGB provided important support for clinicians to make accurate treatment decisions.

## Figures and Tables

**Figure 1:** The plot of the LASSO model: (a) optimal parameter (*λ*) selection in the LASSO model, with the optimal tuning parameter log (*λ*) in the horizontal coordinate and the regression coefficients in the vertical coordinate; (b) distribution of LASSO coefficients about the clinical factors, with the optimal tuning parameter log (*λ*) in the horizontal coordinate and the binomial deviation in the vertical coordinate.

**Figure 2:** The correlation heat map of risk factors.

**Figure 3:** The plot of 10-fold cross-validation. LR: logistic regression; GBM: gradient boosting machine; XGB: extreme gradient boosting; RF: Random Forest; DT: Decision Tree; NBC: Naïve Bayesian model.

**Figure 4:** Feature importance distribution map of ML models.

**Figure 5:** The risk web calculator was designed based on the GBM model.

**Table 1:** Univariate and multivariate logistic regression for the risk of bone metastasis in patients with renal cancer.

Characteristics	Univariate logistic regression			Multivariable logistic regression		
	OR	CI	*P*	OR	CI	*P*
Brain metastases						
No	Ref	Ref	Ref	Ref	Ref	Ref
Yes	14.72	12.24-17.7	<0.001	2.46	1.98-3.05	<0.001
Grade						
Well differentiated						
Moderately differentiated	1.89	1.14-3.13	0.014	1.62	0.97-2.69	0.064
Poorly differentiated	5.84	3.57-9.56	<0.001	3.08	1.87-5.08	<0.001
Undifferentiated; anaplastic	13.92	8.48-22.84	<0.001	4.47	2.69-7.42	<0.001
Unknown	21.09	13.05-34.09	<0.001	7.97	4.9-12.97	<0.001
Liver metastasis						
No	Ref	Ref	Ref	Ref	Ref	Ref
Yes	15.57	13.54-17.9	<0.001	2.37	2.01-2.8	<0.001
N						
N0	Ref	Ref	Ref	Ref	Ref	Ref
N1	10.08	8.99-11.3	<0.001	2.18	1.9-2.51	<0.001
N2	4.47	2.88-6.94	<0.001	1.58	0.97-2.58	0.067
NX	4.88	4.14-5.75	<0.001	1.64	1.34-2.01	<0.001
Pulmonary metastasis						
No	Ref	Ref	Ref	Ref	Ref	Ref
Yes	18.6	16.8-20.61	<0.001	5.2	4.58-5.89	<0.001
T						
T1	Ref	Ref	Ref	Ref	Ref	Ref
T2	4.53	3.93-5.23	<0.001	2.13	1.81-2.5	<0.001
T3	3.78	3.34-4.27	<0.001	1.84	1.59-2.13	<0.001
T4	10.76	9-12.88	<0.001	2.08	1.68-2.59	<0.001
TX	18.08	15.14-21.59	<0.001	3.11	2.51-3.86	<0.001

## Data Availability

The training group data analyzed in this study are from the SEER database (http://seer.cancer.gov/about/), where the analysis of anonymous data is exempt from medical ethics review and does not require informed consent from patients.

## Abbreviations

BM: Bone metastasis
RCC: Renal cell carcinoma
ML: Machine learning
SEER: Surveillance, Epidemiology, and End Results
LR: Logistic regression
GBM: Gradient boosting machine
XG: Extreme gradient boosting
RF: Random Forest
DT: Decision Tree
NBC: Naive Bayesian model
AUC: Area under the curve
mRCC: Metastatic RCC
SER: Skeletal-related events
OST: Overall survival time
PDF: Probability density functions
CUC: Clinical utility curves
MSKCC model: Memorial Sloan Kettering Cancer Center-based poor-risk groups
IMDC model: International Metastatic Renal Cell Carcinoma Database Consortium-based poor-risk groups
GRCC model: Gustave Roussy Cancer Campus
B-FOM scoring system: Fujimoto–Owari–Miyake bone score
TGF-*β*: Transforming growth factor-*β*
FGF: Fibroblast growth factor.
